The article "Multifactor Analysis and Intervention Study on Menstrual Disorders of Female Athletes in the Context of the Winter Olympic Games: A Case-Control Study Based on a Large Sample" was retracted in 2023. Reasons: unreliable results or conclusions; concerns about the data; concerns about the results or conclusions; concerns about the peer review.

# Multifactor Analysis and Intervention Study on Menstrual Disorders of Female Athletes in the Context of the Winter Olympic Games: A Case-Control Study Based on a Large Sample

**DOI:** 10.1155/2022/2985557

**Published:** 2022-05-14

**Authors:** Yuhong Zhang, Xinyue Lu, Longying Wang, Min An, Xibin Sun

**Affiliations:** ^1^1 The First Affiliated Hospital of Hebei North University Department of Obstetrics and Gynecology, Hebei, Zhangjiakou 075000, China; ^2^2 The First Affiliated Hospital of Hebei North University Department of Laboratory Medicine, Hebei, Zhangjiakou 075000, China

## Abstract

A case-control study was conducted to explore the multifactor analysis and intervention of menstrual disorders in female athletes under the background of the Winter Olympic Games, which is based on a large sample. For this purpose, from January 2020 to September 2021, 381 female athletes in long-term ice and snow sports were investigated by random sampling. All of them promoted gynecological examination and counted the incidence of menstrual disorders. The subjects were assigned into two groups according to their menstrual status: abnormal (*n* = 163) and normal menstrual state groups (*n* = 218). The basic and clinical data of the two groups were compared, and univariate analysis and multivariate logistic regression analysis were employed to explore the risk factors of menstrual disorders in female athletes. According to the random number table method, the menstrual disorder group was again assigned into the intervention group and the control group. The intervention group received health education and glucose supplement intervention to correct EAMDs, while the control group only received health education. The improvement of patients' ability balance and the changes of reproductive hormones were compared after intervention. The results of univariate analysis indicated that there exhibited no significant differences in age, menarche age, smoking history, drinking history, grade, sexual life history, abortion history, BMI, and location of household registration, but there were significant differences in family history, sleep quality, diet regularity, and mental health status (*P* < 0.05). The results of univariate analysis indicated that there exhibited no significant differences in age, menarche, smoking, drinking, grade, sexual life history, abortion history, family history, sleep quality, diet regularity, and mental health status. Logistic regression analysis indicated that family history of menstrual disorders, poor sleep quality, irregular diet, and mental health status all affected women's menstrual disorders (OR: 1.411, 95% CI: 1.378∼1.444; OR: 1.501, 95% CI: 1.030∼2.187; OR: 1.554, 95% CI: 1.086∼2.225; OR: 1.383, 95% CI: 1.018∼1.877, respectively) independent risk factors. According to the comparison of menstrual cycle, in the intervention group, 12 patients had menstrual cycle 21–28 days, 12 patients had menstrual cycle 28–38 days, and 58 patients were irregular and had no amenorrhea, while in the control group, 36 patients had menstrual cycle 21–28 days, 24 patients had 28–38 days, 12 patients had amenorrhea, and 11 patients had irregular menstruation, and there exhibited no significant difference (*P* > 0.05). There exhibited no significant difference in energy balance before and after intervention (*P* > 0.05); after intervention, the ability balance of the two groups was significantly promoted, and the degree of improvement in the study group was better (*P* < 0.05). The indexes of reproductive hormones in the follicular phase were compared before and after glucose supplement intervention, and there exhibited no significant difference before intervention (*P* > 0.05); after intervention, the serum LH and GnRH of the two groups decreased, while FSH and P increased. The improvement degree of the intervention group was better than that of the control group, but there exhibited no significant difference (*P* > 0.05). Before intervention, there exhibited no significant difference in the serum E2 level in the follicular phase (*P* > 0.05); after the intervention, the serum E2 of the two groups increased significantly, and the improvement of the intervention group was better (*P* < 0.05). Before intervention, there exhibited no significant difference in the serum E2 level in the follicular phase (*P* > 0.05); after the intervention, the serum E2 of the two groups increased significantly, and the improvement of the intervention group was better (*P* < 0.05). Before intervention, there exhibited no significant difference in serum E2 and P levels in the luteal phase (*P* > 0.05); after intervention, the level of serum E2 decreased and the level of serum P increased in the two groups. There exhibited no significant difference in the level of serum E2 (*P* > 0.05). There exhibited significant difference in the serum P level (*P* < 0.05). Female athletes have a high rate of menstrual disorders. Family history of menstrual disorders, poor sleep quality, irregular diet, and poor mental health are the main risk factors of menstrual disorders. Health education and sugar supplement intervention measures for female athletes play a positive role in the improvement of their ability balance and the regulation of reproductive hormones.

The article "Multifactor Analysis and Intervention Study on Menstrual Disorders of Female Athletes in the Context of the Winter Olympic Games: A Case-Control Study Based on a Large Sample" was retracted in 2023. Reasons: unreliable results or conclusions; concerns about the data; concerns about the results or conclusions; concerns about the peer review.

## 1. Introduction

Exercise-induced menstrual disorder (EAMD) is a special medical problem that perplexes female athletes and coaches, including exercise-induced amenorrhea (AA), sparse menstruation, anovulatory cycle, and luteal insufficiency (LPD) [1]. According to the severity of EAMDs, the order from severe to mild was amenorrhea, sparse menstruation, anovulatory cycle, and LPD [2]. Although exercise-induced amenorrhea is the most serious form of menstrual disorders, other forms of menstrual disorders can also lead to lower levels of estrogen and progesterone and affect the health, bone health, and fertility of athletes [3].

A menstrual cycle is defined as the first day of menstruation to the day before the next menstrual cycle and is usually 21–35 days. Likewise, the menstrual period usually lasts 3–7 days as described in literature [4]. There are primary and secondary amenorrhea: primary amenorrhea refers to the postponement of menarche (normal development of secondary sexual characteristics but no menstruation at the age of 15 or chest development before the age of 10 but no menstruation within 5 years after development) [5]. Secondary amenorrhea refers to menarche but no menstruation for more than 90 consecutive days. Sparse menstruation refers to the extension of the menstrual cycle to 36–90 days [6]. Anovulation refers to anovulation caused by low secretion of luteinizing hormone (LH) and follicle-stimulating hormone (FSH), resulting in decreased levels of estrogen and lack of progesterone [7]. Luteal insufficiency refers to ovulation in the menstrual cycle, but luteal secretion of progesterone is insufficient or the corpus luteum prematurely declines luteal dysfunction, so that the endometrium cannot be converted in time, affecting the implantation of fertilized eggs [8].

Relatively serious menstrual cycle disorders (amenorrhea and sparse menstruation) can be found through follow-up observation and questionnaire survey, while the lighter forms of menstrual cycle disorders (anovulation and luteal dysfunction) need to employ laboratory or clinical diagnostic methods to understand their follicular development and hormone activity [9]. Many athletes with regular menstrual cycle often have the problems of prolonged follicular period, shortened luteal phase, or low progesterone level. For sports researchers and medical supervisors, ovulation can be monitored by tracking changes in LH and progesterone (or their metabolites) in blood or urine. The peak concentration of progesterone in the anovulatory cycle was ≤5 ng/ml, and no peak of serum LH was observed in the middle stage of menstrual cycle [10]. Usually, ovulation of mature follicles occurs within 24 hours after the appearance of LH peak. In addition, we can also observe the basal body temperature (BBT) to understand the ovarian function of athletes. BBT reflects the level of energy metabolism of the body in a resting state. In women with normal ovarian function, the daily basic body temperature of a menstrual cycle is recorded on the basic body temperature sheet, and the curve is biphasic, that is, the biphasic body temperature curve, the BBT of the follicular phase is lower, and the body temperature of the luteal phase after ovulation is 0.3–0.5°C higher compared with the first half of the ovulation. This is because the progesterone produced by the luteum in the second half of the cycle acts on the hypothalamic thermoregulation center and the BBT increases slightly. If BBT is monophasic, there is no increase in body temperature in the second half of the menstrual cycle, indicating that there is no luteal formation and lack of progesterone in this cycle, so the monophasic body temperature curve indicates that the cycle is anovulatory. The two-way temperature cycle does not necessarily indicate ovulation because, in some menstrual cycles, when the follicle is mature but not ruptured, the egg cells are not excreted, but the granulosa cells are still luteinized to form the luteal corpus luteum and secrete progesterone, which is called “unruptured follicular luteinization syndrome” [11]. Only based on basic body temperature measurement cannot accurately monitor the occurrence of ovulation; hence, the basic body temperature method can be used in combination with hormone detection or B-ultrasound monitoring, and it can strengthen the accuracy of ovulation monitoring.

The article "Multifactor Analysis and Intervention Study on Menstrual Disorders of Female Athletes in the Context of the Winter Olympic Games: A Case-Control Study Based on a Large Sample" was retracted in 2023. Reasons: unreliable results or conclusions; concerns about the data; concerns about the results or conclusions; concerns about the peer review.

The causes of menstrual disorders in EAMDs have been the focus of research and attention of scholars, and a variety of factors can have a certain impact on the menstrual status of patients [12]. Therefore, it is necessary to investigate and study the menstrual disorders of women of childbearing age, especially female athletes, monitor their menstrual status, and explore the main influencing factors of menstrual disorders, which play an important role in improving the physiological health status of female athletes [13].

In this paper, we have presented a naïve approach to resolve these issues associated with the existing state of the art approaches. For this purpose, we have collected data related to 381 long-term ice and snow sports female athletes specifically those who are treated in our hospital from January 2020 to September 2021. Initially, these patients or athletes were divided into two different groups, i.e., normal mental state and abnormal mental state groups. These patients were evaluated for mental disorder by utilizing the proposed methodology. Moreover, age factor were considered while making these groups.

The article "Multifactor Analysis and Intervention Study on Menstrual Disorders of Female Athletes in the Context of the Winter Olympic Games: A Case-Control Study Based on a Large Sample" was retracted in 2023. Reasons: unreliable results or conclusions; concerns about the data; concerns about the results or conclusions; concerns about the peer review.

The rest of the manuscript is organized as follows.

In the subsequent section, a detailed description of patient's selection criteria and evaluation is presented. Moreover, treatment and observation mechanisms were described. Results of the experimental studies, which were carried out during the proposed setup, are presented in Section 3 of the paper. Finally, concluding remarks are given.

## 2. Patients and Methods

In this section, we are going to describe how patients were selected and how they are divided into various groups.

### 2.1. General Information

Three hundred and eighty-one (381) female athletes in long-term ice and snow sports, specifically from January 2020 to September 2021, were investigated and analyzed through the random sampling technique. All of them promoted gynecological examination and counted the incidence of menstrual disorders. The subjects were assigned into two groups according to their menstrual status: abnormal menstruation group (*n* = 163) and normal menstrual state group (*n* = 218). In the menstrual disorder group, the age was 17–26 years old, with an average of (22.43 ± 3.21) years, and the age of menarche was 11–15 years old, with an average of (13.25 ± 2.07) years old. In the normal menstruation group, the age of menarche was (22.91 ± 3.44) years old, and the age of menarche was 11 years old, with an average age of (13.66 ± 2.13) years. There was no statistical significance in the general data. This study was permitted by the Medical Ethics Association of our hospital, and all patients noticed informed consent.

#### 2.1.1. Selection Criteria

- Negative energy balance
- Female athletes over 17 years old
- Suffering from exercise-induced menstrual cycle disorder

Exercise-induced menstrual cycle disorders include delayed menarche, sparse menstruation, short menstrual cycle (short corpus luteum and luteal dysfunction) or too long, low menstrual volume, low estrogen and progesterone, anovulatory menstrual cycle, and amenorrhea.

#### 2.1.2. Exclusion Criteria

1. Positive energy balance
2. Hyperprolactinemia
3. Polycystic ovary syndrome
4. Thyroid diseases (hyperthyroidism, hypothyroidism, etc.)
5. Recently taken various hormone drugs

### 2.2. Treatment Methods

#### 2.2.1. Questionnaire Survey of Menstrual Disorders

All the subjects received a unified questionnaire, a self-made questionnaire, which included name, age, location of household registration, class, smoking history, drinking history, age of menarche, BMI, sexual life history, abortion history, family history of menstrual disorders, sleep quality, diet regularity, mental health status, menstrual physical status, and so on. According to the information of the questionnaire, the occurrence of menstrual disorders was counted and the incidence of menstrual disorders was calculated. Menstrual disorder criteria: when the subjects have menstrual cycle or blood loss disorder, the menstrual period can be accompanied by premenstrual, menstrual abdominal pain. According to menstrual status, menstrual disorders were assigned into menstrual disorders group and normal menstruation group. The basic and clinical data of the two groups were compared, and the above-mentioned indexes of the two groups were analyzed by univariate analysis. A logistic multiple regression model of menstrual disorders was established to analyze and explore the risk factors of menstrual disorders in female athletes.

The article "Multifactor Analysis and Intervention Study on Menstrual Disorders of Female Athletes in the Context of the Winter Olympic Games: A Case-Control Study Based on a Large Sample" was retracted in 2023. Reasons: unreliable results or conclusions; concerns about the data; concerns about the results or conclusions; concerns about the peer review.

#### 2.2.2. Intervention Method

Carrying out the health education intervention to the normal menstruation group, the main intervention contents are as follows:

1. Carry out the psychological intervention to the patients in the disorder group, communicate actively with the patients, shorten the distance with the patients by way of conversation, carry on the psychological counseling to them, improve the bad psychological mood of the patients, especially the anxiety, depression, irritability, and other emotions caused by menstrual disorders, and make the patients maintain a positive and optimistic state of mind
2. Carry out gynecological health education intervention for patients to explain the knowledge of menstruation and matters needing attention during menstruation, such as avoiding cold water during menstruation, avoiding raw and cold food, and paying attention to rest and cleanliness
3. Guidance of daily life, guidance and intervention on patients' daily activities, so as to form a good regular sleep time, eat regularly for three meals a day, pay attention to reasonable dietary collocation, supplement daily nutritional needs, strengthen physical exercise, reduce bad habits in daily life, and so on
4. The intervention group added oligosaccharide supplement intervention on the basis of the control group, and the specific methods are as follows: the sugar used in this study is “Lidi strong oligosaccharide solid beverage,” which is mainly composed of maltose oligosaccharides, which is provided by Shanghai Litong Biochemical Products Co., Ltd., product implementation standard: GB7101-2003, food production license number: QS311406010048, and passed the test of China Doping Testing Center. It was included in the list of Sports Nutrition products of Shanghai Sports Bureau in 2012.

The sports beverage ingredients mainly include maltose oligosaccharides, crystal fructose, fish protein meal, sodium chloride, and so on; 75 g per bag, 62 g maltose oligosaccharides and 10 g fructose. After energy conversion, it is concluded that each bag of sugar can provide energy of about 287 Kcal. The main results are as follows:

(1) *The formulation of the amount of sugar supplement*: the weighing method was employed to mobilize the diet survey of three meals, and the bookkeeping method was employed in the survey of snacks other than three meals. In this experiment, during the 3–9 days of the early follicular stage, the daily food intake of the subjects was recorded or observed for seven (7) consecutive days. After the conversion of the raw-to-cooked ratio of the food weighing value, all the data were entered into the Jian Dian software automatic Food King 7.0, and the results of dietary analysis were obtained. While taking part in the dietary survey, the subjects wore the SenseWear Armband energy monitoring table produced by BodyMedia Company in the United States, recorded the daily energy consumption in these 7 days and analyzed the athletes' energy consumption using SenseWearProfessional7.0 software. As a result, the daily energy intake and energy consumption of the subjects were obtained for one week (six training days and one rest day). By calculating the average value of the difference between daily energy intakes minus daily energy consumption, the energy balance of each subject is reflected. According to the energy value provided by each bag of sports drinks, the number of bags of sugar drinks that each subject should supplement is calculated in order to restore the energy balance of athletes (energy intake is equal to energy consumption) and achieve the purpose of increasing their available energy. (2) *Sugar supplement*: the supplement of oligosaccharide solid beverage is during each training period from Monday to Saturday, from the early follicular stage of the first menstrual cycle to the end of the middle luteal phase of the third menstrual cycle (the last blood collection). The actual duration is about 3 menstrual cycles. According to the training arrangement of the coaches, the researchers prepared the sports drinks in proportion according to the beverage instructions, supervised and instructed the athletes to supplement according to the prescribed amount in the process of sports training, and urged them to ensure a normal diet every day.

The article "Multifactor Analysis and Intervention Study on Menstrual Disorders of Female Athletes in the Context of the Winter Olympic Games: A Case-Control Study Based on a Large Sample" was retracted in 2023. Reasons: unreliable results or conclusions; concerns about the data; concerns about the results or conclusions; concerns about the peer review.

### 2.3. Observation Index

#### 2.3.1. Physical Basic Condition Test

The height, weight, and body fat rate of all subjects were measured before and after the intervention of glucose supplementation for about 3 menstrual cycles. The height and weight were measured by TANITA height and weight meter made in Japan, and the body composition was measured by Lunar Prodigy dual energy X-ray absorptiometry produced by GE Company.

#### 2.3.2. Menstrual Disorder Blood Test

The time of blood collection was arranged at 14 ± 2 days (late follicular stage) and 22 ± 2 days (mid-luteal phase) of one menstrual cycle before glucose supplement intervention and at the corresponding time point of the third menstrual cycle before glucose supplement intervention. Blood samples were harvested on the 14th day of the menstrual cycle and around the 22nd day of the menstrual cycle because of the peak secretion of LH, E2, and P hormones, which is helpful for us to observe the changes of hormones. On the day of blood collection, athletes are required to have an empty stomach and no strenuous physical exercise. A total of 8 ml blood was drawn from the median vein of forearm elbow by professional nurses and placed in two coagulation-promoting tubes with each 4 ml in each tube. The extracted blood was placed in 30 min, and a tube of blood was centrifuged at 2500 rpm at room temperature for 20 minutes. 1 ml serum was taken in an EP tube and stored at −80°C for the detection of FSH, estradiol (E2), and progesterone (P); and another tube of blood was centrifuged at 4°C for 20 minutes at 2500 rpm. A total of 600 *μ*l serum was harvested in the EP tube and stored at −80°C for detection of LH and gonadotropin-releasing hormone (GnRH). In order to reduce the batch error, all the blood samples are stored in the refrigerator at −80°C and tested uniformly after the final collection. FSH, E2, and P were determined by immunochemiluminescence (ICMA). *Reagent*: FSH, E2, and P immune chemiluminescence kits produced by Beckman Coulter Co., Ltd. *Detection instrument*: the fully automatic chemiluminescence immunoassay system Access2 immunoassay system produced by Beckman Coulter Co., Ltd. GnRH and LH were determined by immunoassay (RIA). *Reagent*: GnRH and LH radioimmunoassay kits provided by the Biblical Biology Department of the Second Military Medical University of the Chinese People's Liberation Army. The main testing instruments are SN695B intelligent counter produced by the Sun Ring instrument Factory of Shanghai Institute of Atomic Energy, Chinese Academy of Sciences, and DL-8 cryogenic centrifuge produced by Shanghai Institute of Centrifugal Machinery. *Auxiliary testing instruments*: B11-2 constant temperature magnetic agitator—Shanghai Siler instrument Co., Ltd.—HH · W21 · 600S digital display electric thermostat, Haier low-temperature refrigerator, Haier incubator refrigerator, and LABCONCO freeze dryer.

### 2.4. Statistical Analysis

SPSS 18.0 statistical software was employed to process and analyze the data of menstrual disorders. The measurement data of homogeneity of variance were expressed by mean ± standard deviation (M ± SD); the comparison between energy metabolism and blood index groups was conducted by the independent-sample t-test, and the paired-sample t-test was employed to compare energy metabolism and blood index groups before and after oligosaccharide supplement intervention. If *P* < 0.05, the difference of dysmenorrhea was significant.

The article "Multifactor Analysis and Intervention Study on Menstrual Disorders of Female Athletes in the Context of the Winter Olympic Games: A Case-Control Study Based on a Large Sample" was retracted in 2023. Reasons: unreliable results or conclusions; concerns about the data; concerns about the results or conclusions; concerns about the peer review.

## 3. Experimental Results

### 3.1. Single-Factor Analysis of Menstrual Disorders

First of all, we analyzed the influencing factors of menstrual disorders; univariate analysis indicated that there exhibited no significant differences in age, menarche age, smoking history, drinking history, grade, sexual life history, abortion history, BMI, location of household registration, but there exhibited significant differences in family history, sleep quality, dietary regularity, and mental health status (*P* > 0.05). All the results are indicated in Table 1.

Table 1 shows the comparison of nursing satisfaction between the two groups [*n*/%].

### 3.2. Logistic Regression Analysis of Influencing Factors of Menstrual Disorders

Through univariate analysis, the relevant indicators with statistical significance were substituted into the logistic model for multifactor analysis. Taking irregular menstruation (defined as “No” = 0, “Yes” = 1) as a dependent variable (Table 2 of assignment table), logistic regression analysis was carried out. The results indicated that family history of menstrual disorders, poor sleep quality, irregular diet, and mental health status all affected female menstrual disorders (OR: 1.411, 95% CI: 1.378∼1.444; OR: 1.501, 95% CI: 1.030∼2.187; OR: 1.554, 95% CI: 1.086∼2.225, OR: 1.383, 95 CI%: 1.018∼1.877, respectively). The detailed results are indicated in Table 3.

### 3.3. Comparison of Basic Conditions between Intervention Group and Control Group

We have compared the basic situation of the two groups, and there exhibited no significant difference in age, height, weight, years of special training, and age of initial training (*P* > 0.05). All the data results are indicated in Table 4.

### 3.4. Comparison of the Menstrual Cycle

According to the comparison of the menstrual cycle, in the intervention group, twelve (12) patients had menstrual cycle 21–28 days, 12 patients had menstrual cycle 28–38 days, and 58 patients had irregular menstruation, whereas in the control group, 36 patients had menstrual cycle 21–28 days, 24 patients had menstrual cycle 28–38 days, 12 patients had amenorrhea, and 11 patients had irregular menstruation. There exhibited no significant difference (*P* > 0.05). All the results are indicated in Figure 1.

The article "Multifactor Analysis and Intervention Study on Menstrual Disorders of Female Athletes in the Context of the Winter Olympic Games: A Case-Control Study Based on a Large Sample" was retracted in 2023. Reasons: unreliable results or conclusions; concerns about the data; concerns about the results or conclusions; concerns about the peer review.

### 3.5. Comparison of Energy Balance between the Two Groups before and after Intervention

We compared the energy balance before and after intervention, and there exhibited no significant difference before intervention (*P* > 0.05). The degree of improvement in the study group was better than that in the control group (*P* < 0.05). All the results are indicated in Table 5.

### 3.6. Comparison of Reproductive Hormone Indexes in Follicular Phase before and after Glucose Supplement Intervention

We compared the indexes of reproductive hormones in the follicular phase before and after glucose supplement intervention, and there exhibited no significant difference before intervention (*P* > 0.05); after intervention, the serum LH and GnRH of the two groups decreased, while FSH and P increased. The improvement degree of the intervention group was better than that of the control group, but with no significant difference (*P* > 0.05). All the results are indicated in Table 6.

Before intervention, there was no significant difference in the serum E2 level in the follicular phase (*P* > 0.05); after the intervention, the serum E2 of the two groups increased significantly, and the improvement degree of the intervention group was better than that of the control group (*P* < 0.05). All the results are indicated in Table 7.

### 3.7. Comparison of Reproductive Hormone Indexes in Luteal Phase of Subjects before and after Glucose Supplement Intervention

We have compared the reproductive hormone indexes of the subjects in the luteal phase before and after glucose supplementation. Before the intervention, there exhibited no significant difference in the level of reproductive hormone (*P* > 0.05); after intervention, the serum LH, GnRH, and FSH of the two groups decreased, and the improvement degree of the intervention group was better than that of the control group (*P* < 0.05). All the results are indicated in Table 8.

Before intervention, there exhibited no significant difference in serum E2 and P levels in the luteal phase (*P* > 0.05); after intervention, the level of serum E2 decreased and the level of serum P increased in the two groups. There exhibited no significant difference in the level of serum E2 (*P* > 0.05). And there exhibited significant difference in the serum P level (*P* < 0.05). All the results are indicated in Table 9.

## 4. Discussion

Exercise-induced menstrual cycle disorders include exercise-induced amenorrhea, sparse menstruation, anovulatory cycle, and luteal dysfunction [10]. According to the severity and EAMD form, the order from severe to mild was amenorrhea, sparse menstruation, anovulatory cycle, and luteal insufficiency [11]. Studies have found that EAMD will lead to abnormal secretion of sex hormones in female athletes, affecting athletes' sports ability, sports career, bone mineral density, and fertility. In medicine, amenorrhea is usually assigned into two forms: primary amenorrhea and secondary amenorrhea. Primary amenorrhea refers to the postponement of the age of menarche; and secondary amenorrhea refers to having menarche but no menstruation for more than three months in a row [12]. Sparse menstruation is only 3 to 4 menstruation a year. Anovulatory menstruation refers to anovulatory menstruation due to the low secretion of LH and FSH, resulting in lack of estrogen and progesterone, but the appearance observation is that there is menstrual bleeding [13]. LPD refers to insufficient secretion of estrogen and progesterone or premature decline of corpus luteum due to lack of endocrine function, resulting in insufficient secretion and transformation of endometrium. The short luteal phase indicates luteal dysfunction, which is not conducive to the implantation of fertilized eggs and is prone to infertility or abortion [14].

The article "Multifactor Analysis and Intervention Study on Menstrual Disorders of Female Athletes in the Context of the Winter Olympic Games: A Case-Control Study Based on a Large Sample" was retracted in 2023. Reasons: unreliable results or conclusions; concerns about the data; concerns about the results or conclusions; concerns about the peer review.

There are many literature studies on the epidemiology of sparse menstruation and amenorrhea in female athletes [15]. The proportion of these two relatively more severe forms of menstrual disorders among runners is 6%–43%, and the proportion of athletes in different sports in high school and college is 1%–31%, which exceeds the observed prevalence rate of ordinary female college students [16]. However, there are few studies on the prevalence of mild forms of menstrual disorders (LPD and anovulation). In 1998, DeSouza et al. investigated 24 runners and 11 sedentary controls with a total of 100 menstrual cycles through daily hormone tests [17]. The subjects had continuous, regular, and normal menstrual cycles. The study found that the prevalence rate of long-distance runners was 48%, of which 79% belonged to LPD and anovulation. Subsequently, in 2010, De Souza et al. conducted a follow-up study report, which was also used to detect hormone metabolites in urine every day [18]. A survey of mild menstrual disorders in patients with normal menstrual cycle found that, in sedentary women, 95.0% (19/20) was normal ovulation and 5.0% (1/20) was luteal insufficiency; and among exercise women, 47.9% (23/48) were normal ovulation, and 52.1% (25/48) were classified as abnormal, of which 27% (13/48) were luteal insufficiency (short and/or inadequate luteal phase) and 25% (12/48) were anovulatory cycles. The prevalence rate of abnormal menstrual cycle in exercise women was much higher than that in sedentary women (*P* < 0.001). For the study of more severe forms of menstrual disorders, it was found that 7.0% (3/43) of exercise women had sparse menstruation and 37.2% (16/43) had amenorrhea, while the control group of sedentary women had no sparse menstruation or amenorrhea [18]. The rate of amenorrhea in exercise women was significantly higher than that in sedentary women (*P* < 0.023). Through the analysis of urinary hormone levels in two consecutive menstrual cycles, Wang et al. discussed the incidence of LPD and anovulation in female athletes with regular menstrual cycles [19]. A total of 30 athletes from different sports (including sprint, medium- and long-distance running, pole vaulting, weightlifting, martial arts, fencing, and taekwondo) were all with abnormal ovarian function; among them, 10 (33.3%) had luteal insufficiency, 8 (26.7%) had anovulatory cycles, and 12 (40.0%) had inconsistent performance before and after two consecutive menstrual cycles. Among the 60 menstrual cycles monitored, there were 2 normal ovulation cycles (3.3%), 32 LPD cycles (53.3%), and 26 anovulatory cycles (43.3%) [20]. The 16 menstrual cycles of 8 normal college students in the control group were normal ovulation cycles. Menstrual disorders are very common among female athletes, the rate of amenorrhea in athletes is much higher than that in ordinary women, and there are differences in the occurrence of menstrual disorders, such as long-distance runners' menstrual cycle prolongation or shortening rate as high as 40%; for long-term endurance sports, the incidence of EAMD is higher [21].

The article "Multifactor Analysis and Intervention Study on Menstrual Disorders of Female Athletes in the Context of the Winter Olympic Games: A Case-Control Study Based on a Large Sample" was retracted in 2023. Reasons: unreliable results or conclusions; concerns about the data; concerns about the results or conclusions; concerns about the peer review.

Athletes' physical fitness is closely related to their performance, especially for ice and snow female athletes, how to strengthen their physical fitness and reduce the impact of long-term ice and snow environment on body function is the focus of athletes and scholars [22]. Menstrual disorder is one of the common gynecological diseases, which has a high incidence in clinic. The incidence of menstrual disorders covers patients of all ages during menstruation, among which women of childbearing age are the most widespread. After the onset of the disease, the patients indicated long-term persistent menstrual cycle disorder, abnormal increase or decrease of menstrual volume, accompanied by abdominal pain and general discomfort before and after menstruation, which seriously affected the normal life of the patients [22, 23]. Menstrual disorder has become a common social problem and has aroused great concern of gynecological clinicians. Therefore, how to reduce the clinical incidence of menstrual disorders has become the main research direction of clinicians. At present, there is a lack of research on the occurrence and current situation of menstrual disorders in ice and snow athletes. The purpose of this study is to analyze the influencing factors of menstrual disorders in long-term ice and snow athletes and to provide effective prevention and intervention measures for female ice and snow athletes.

The article "Multifactor Analysis and Intervention Study on Menstrual Disorders of Female Athletes in the Context of the Winter Olympic Games: A Case-Control Study Based on a Large Sample" was retracted in 2023. Reasons: unreliable results or conclusions; concerns about the data; concerns about the results or conclusions; concerns about the peer review.

The results of this study indicated that there were 163 patients with menstrual disorders of varying degrees, with an incidence of menstrual disorders of 42.78%, indicating that the menstrual health status of female athletes was worrying, and the prevention and treatment situation was grim, which should be highly concerned by clinicians [24]. In the univariate analysis of influencing factors, there was no significant difference in age, menarche age, smoking history, drinking history, grade, sexual life history, abortion history, BMI, and household registration between the two groups. The incidence of family history of menstrual disorders, poor sleep quality, irregular diet, and poor mental health in the menstrual disorder group was higher than those in the normal menstruation group. Further multivariate analysis indicated that the family history of menstrual disorders, poor sleep quality, irregular diet, and poor mental health status were the risk factors of menstrual disorders in female athletes. The reason for the analysis is that there is a certain family genetic history of menstrual disorders, and the symptoms related to irregular menstruation in the mother may be inherited to the next generation, with a certain genetic tendency, but its genetic mechanism remains to be further studied. Good sleep is the necessary guarantee of the normal living state of the body. If the sleep quality of the patient is poor, such as short sleep time, staying up late, and insomnia, it is difficult for the patient to get enough rest. It has adverse effects on the patient's mental state and endocrine system and then increases the incidence of menstrual disorders. Therefore, in menstruation and daily life, sleep quality should be improved to ensure adequate sleep time [25]. At present, in order to complete the training goals, female athletes are prone to irregular diet, such as irregular meal time, excessive dieting, and eating spicy and irritating food, which will cause menstrual disorders in patients' living conditions. Spicy stimulating raw and cold food will directly affect the patient's menstrual status. Therefore, the majority of female athletes should eat regularly and adjust their diet structure. Mental health status is also the main factor affecting menstrual disorders. Long-term mental depression, tension, or suffering from major mental stimulation and psychological trauma will affect the endocrine system of patients and have adverse effects on the function of hypothalamus and pituitary, affect the secretion of estrogen in patients, and then exhibit the symptoms of irregular menstruation. Therefore, patients should adjust their psychological state during the menstrual period and maintain a positive and optimistic attitude at all times.

The article "Multifactor Analysis and Intervention Study on Menstrual Disorders of Female Athletes in the Context of the Winter Olympic Games: A Case-Control Study Based on a Large Sample" was retracted in 2023. Reasons: unreliable results or conclusions; concerns about the data; concerns about the results or conclusions; concerns about the peer review.

The main ingredient of sugar beverage employed in this experiment is maltose oligosaccharide [26]. Maltose oligosaccharides have low osmotic pressure (menstrual disorders of glucose 1P4), low sweetness (about 40% of menstrual disorders of sucrose), are absorbed and utilized more slowly than monosaccharides and disaccharides and can provide energy replenishment for the body for a longer time; meanwhile the insulin and blood glucose reactions are relatively stable and do not form fat deposits [24, 25]. This study found that the body weight and body fat rate of long-term ice and snow athletes are basically in the normal range, which may be related to the fact that the project emphasizes the characteristics of endurance and strength quality. In peacetime training, coaches pay attention to the cultivation of endurance, agility, and strength quality but do not emphasize the slimness of physique. After 3 months of glucose supplement intervention, the body weight and body fat rate of athletes did not change significantly, which proved that sugar supplement intervention did not cause fat accumulation and obesity of athletes. As can be seen from the results of the study, the energy of both the intervention group and the control group tended to be positively balanced, and the control group did not experience the intervention of sugar drinks for three months. The reason may be that our control group also carried out health education. To some extent, the control group subjects also supervised and monitored their own reasonable diet. Although the control group improved after three months, it still indicated a negative energy balance. The difference of intragroup comparison was not statistically significant. The intervention group successfully promoted the transition from negative energy balance to positive energy balance during the three-month glucose supplement process and had statistical significance, which demonstrates that glucose supplement intervention is effective to correct the subjects' negative energy balance.

GnRH is a kind of polypeptide hormone secreted by hypothalamic GnRH neurons [25]. The neural network integrates various internal and external factors and steroid hormone levels to control the release of GnRH. The neuroendocrine cells in the hypothalamus synthesize GnRH, which is then released into the blood through the pituitary portal system and transported to the adenohypophysis to promote the secretion of gonadotropins FSH and LH [26]. Gonadotropins reach the gonad through blood circulation, which regulates the secretion of estrogen and progesterone in the ovary and acts on the target organs. The realization of reproductive function depends on the good endocrine environment of the target organs [27]. There are positive and reverse regulation and self-regulation among the hypothalamus, pituitary, and gonad, so as to control and maintain the stability of sex hormone levels and internal environment. FSH and LH are glycoprotein hormones secreted by adenohypophysis, which are regulated by GnRH and sex hormones and change periodically with the menstrual cycle [28]. GnRH-LH pulse indicated low amplitude and high frequency in the late follicular phase and low frequency and high amplitude type in the luteal phase, while FSH had no obvious pulse fluctuation, its half-life was relatively long, and its blood concentration was low [29]. FSH is an essential hormone in the process of follicular development, and its main physiological functions are to promote follicular maturation and promote the secretion of estrogen and progesterone. FSH was at a low level in the early follicular stage, decreased slightly in the late follicular stage, and reached a low value at 24 hours before ovulation, then increased immediately. Together with LH, it decreased 24 hours later and maintained a low level throughout the luteal phase. If the secretion of FSH is insufficient in the follicular phase, it will make the follicular dysplasia and prolong the follicular phase, while the insufficient secretion of FSH in the luteal phase will affect the effect of aromatase in luteal cells. The main physiological function of LH is to promote ovulation and corpus luteum development and maturation. In women of childbearing age, the level of LH in the follicular stage is low, and there is a steep peak before ovulation to trigger ovulation, while a small peak often occurs in the middle luteal phase to maintain luteal function. An abnormal LH/FSH ratio can also cause disorder of gonadal axis function, follicular dysplasia, and luteal hypoplasia after ovulation, resulting in insufficient endometrial secretion response [28].

The article "Multifactor Analysis and Intervention Study on Menstrual Disorders of Female Athletes in the Context of the Winter Olympic Games: A Case-Control Study Based on a Large Sample" was retracted in 2023. Reasons: unreliable results or conclusions; concerns about the data; concerns about the results or conclusions; concerns about the peer review.

E2 is the most bioactive estrogen in women [30]. The content of E2 in the circulating blood of normal women of childbearing age changes periodically: the lowest level in early follicle and the highest in ovulation period, which can reach more than 1800 pmol/L. Progesterone (P) is the main bioactive progesterone secreted by the ovary. The level of progesterone in normal women of childbearing age was lower compared with 2.0 nmol/L before ovulation and higher compared to 8 nmol/L after ovulation. Persistent progesterone levels below 8 nmol/L often indicate ovulation disorders. Clinically, blood samples are usually harvested one week before menstruation, and the ovulation and luteal function of patients are judged according to the results of progesterone concentration determination [29]. Postmenopausal estradiol and progesterone levels are low. EAMDs, especially severe menstrual disorders, are often deficient in estrogen and progesterone secretion. Cui Liping through the detection of saliva E2 and P in one menstrual cycle found that the average levels of E2 and P in the long- and short-menstrual cycle group were significantly lower than those in the control group, especially in the long-cycle group, the hormone level was close to that of amenorrhea [30]. This study found that after the intervention, the serum LH and GnRH of the two groups decreased, while the FSH and P increased. The improvement degree of the intervention group was better. Before the intervention, there was no significant difference in the serum E2 level in the follicular phase; after the intervention, the serum E2 levels increased significantly, and the improvement degree of the intervention was better. Before the intervention, there exhibited no significant difference in the serum E2 level in the follicular phase; after the intervention, the serum E2 levels in the two groups increased significantly, and the improvement degree of the intervention was better. Before the intervention, there exhibited no significant difference in the levels of serum E2 and P. After the intervention, the level of serum E2 decreased and the level of serum P increased. There exhibited no significant difference (*P* > 0.05). And there exhibited significant difference in the serum P level (*P* < 0.05). This demonstrates that sugar supplement is beneficial to improve and restore exercise-induced menstrual cycle disorder.

## 5. Conclusion

In this paper, we have presented a naïve approach to resolve these issues associated with the existing state-of-the-art approaches. For this purpose, we have collected data related to 381 long-term ice and snow sports female athletes specifically those who are treated in our hospital from January 2020 to September 2021. Initially, these patients or athletes were divided into two different groups, i.e., normal mental state and abnormal mental state groups. These patients were evaluated for mental disorder by utilizing the proposed methodology. Moreover, age factor were considered while making these groups. Finally, the incidence of EAMDs in female athletes is high, and there is a widespread negative energy balance. For female athletes with menstrual disorders, relevant health education intervention measures should be taken, and oligosaccharide supplements should be given if necessary, which can facilitate the recovery of reproductive hormone levels of athletes with sports menstrual cycle disorders and improve the levels of serum E2 in the serum follicular phase and serum P in the luteal phase.

The article "Multifactor Analysis and Intervention Study on Menstrual Disorders of Female Athletes in the Context of the Winter Olympic Games: A Case-Control Study Based on a Large Sample" was retracted in 2023. Reasons: unreliable results or conclusions; concerns about the data; concerns about the results or conclusions; concerns about the peer review.

## Figures and Tables

**Figure 1:** Menstrual cycle of two groups of subjects.

**Table 1:** Single-factor analysis of menstrual disorders.

Related factors	Menstrual disorder group (*n* = 163)	Normal menstruation group (*n* = 218)	*t*/*χ*2	*P*
Age (years)	22.43 ± 3.21	22.91 ± 3.44	1.386	>0.05
Age of menarche (age)	13.25 ± 2.07	13.66 ± 2.13	1.881	>0.05
BMI (kg/m^2^)	21.93 ± 2.75	22.14 ± 2.88	0.718	>0.05
Smoking history (*n*/%)			1.199	>0.05
Yes	4 (2.45)	10 (4.59)		
None	159 (97.55)	208 (95.41)		
Drinking history (*n*/%)			2.190	>0.05
Yes	7 (4.29)	55 (25.23)		
None	156 (95.71)	163 (30.73)		
Training years			0.683	>0.05
<1 Year	40 (24.54)	61 (27.98)		
1∼3 Year	51 (31.29)	65 (29.81)		
3∼8 Year	38 (23.31)	51 (23.39)		
>8 Year	34 (20.86)	41 (18.81)		
Sexual life history			0.059	>0.05
Yes	52 (31.90)	67 (30.734)		
None	111 (68.10)	151 (69.27)		
History of flow of people			0.003	>0.05
Yes	11 (6.75)	15 (6.88)		
None	152 (93.25)	203 (93.12)		
Family history of menstrual disorders			12.576	<0.01
Yes	75 (46.01)	140 (64.22)		
None	88 (53.99)	78 (35.78)		
Sleep quality			27.773	<0.01
Good	54 (33.13)	126 (57.80)		
Poor	109 (66.87)	92 (42.20)		
Dietary regularity			75.265	<0.01
Law	56 (34.36)	171 (78.44)		
Irregular	107 (65.64)	47 (21.56)		
Mental health status			102.331	<0.01
Good	83 (50.92)	208 (95.41)		
Poor	80 (49.08)	10 (4.59)		

**Table 2:** Logistic regression analysis variable assignment table.

Classification	Variable	Assignment	
Dependent variable	Menstrual disorder	None = 0	Yes = 1
Independent variable	Family history of menstrual disorders	Yes = 1	None = 0
	Sleep quality	Difference = 1	Good = 0
	Irregular diet	Yes = 1	None = 0
	Psychological condition	Difference = 1	Good = 0

**Table 3:** Logistic regression analysis of influencing factors of menstrual disorder.

Project	*β* value	SE	Wald value	*P* value	OR value (95% CI)
Family history of menstrual disorders	0.344	0.012	821.778	<0.001	1.411 (1.378∼1.444)
Poor sleep quality	0.406	0.192	4.471	<0.05	1.501 (1.030∼2.187)
Irregular diet	0.441	0.183	5.807	<0.05	1.554 (1.086∼2.225)
Mental health status	0.324	0.156	4.314	<0.05	1.383 (1.018∼1.877)

**Table 4:** Comparison of basic conditions between intervention group and control group [$\bar{x}\pm s$].

Group	*N*	Age (years)	Height (cm)	Body weight (kg)	Number of years of special training (years)		Age of initial training (years)
Intervention group	81	20.74 ± 2.45	166.23 ± 8.03	56.84 ± 8.41		3.41 ± 3.05	13.71 ± 3.24
Control group	82	21.32 ± 3.03	166.07 ± 3.62	58.17 ± 9.29		3.53 ± 2.23	13.24 ± 2.31
*t*		1.343	0.164	0.958		0.287	−1.067
*P*		>0.05	>0.05	>0.05		>0.05	>0.05

The article "Multifactor Analysis and Intervention Study on Menstrual Disorders of Female Athletes in the Context of the Winter Olympic Games: A Case-Control Study Based on a Large Sample" was retracted in 2023. Reasons: unreliable results or conclusions; concerns about the data; concerns about the results or conclusions; concerns about the peer review.

**Table 5:** Comparison of energy balance between the two groups before and after intervention [$\bar{x}\pm s$].

Group	*N*	Capacity balance		*t*	*P*
		Before intervention	After intervention		
Intervention group	81	−467.91 ± 367.12	123.54 ± 107.78	13.912	<0.05
Control group	82	−445.66 ± 305.78	−188.42 ± 195.65	6.417	
*t*		0.421	12.578		
*P*		>0.05	<0.05		

**Table 6:** Comparison of LH, GnRH, and FSH levels in the follicular phase of subjects before and after glucose supplement intervention [$\bar{x}\pm s$].

Group	*N*	LH (mIU/ml)		GnRH (pg/ml)		FSH (mIU/ml)	
		Before intervention	After intervention	Before intervention	After intervention	Before intervention	After intervention
Intervention group	81	12.61 ± 4.53	11.62 ± 2.14	38.45 ± 37.01	33.51 ± 24.45	5.13 ± 2.75	6.63 ± 1.64
Control group	82	13.47 ± 4.91	12.13 ± 2.08	47.73 ± 36.84	40.73 ± 33.61	5.34 ± 1.76	6.56 ± 1.92
*t*		1.162	0.787	1.604	1.566	0.581	0.250
*P*		>0.05	>0.05	>0.05	>0.05	>0.05	>0.05

**Table 7:** Changes in E2 and *P* indexes in the follicular phase before and after glucose supplement intervention [$\bar{x}\pm s$].

Group	*N*	E2 (pg/ml)		*P* (ng/ml)		
		Before intervention	After intervention	Before intervention	After intervention	
Intervention group	81	52.44 ± 6.53	88.54 ± 41.13	0.92 ± 0.21	1.04 ± 0.33	
Control group	82	51.18 ± 8.26	36.74 ± 9.26	1.01 ± 1.34	1.11 ± 0.31	
*t*		1.080	11.123	0.597	1.396	
*P*		>0.05	<0.05	>0.05	>0.05	

**Table 8:** Comparison of LH, GnRH, and FSH levels in the luteal phase of subjects before and after glucose supplementation [$\bar{x}\pm s$].

Group	*N*	LH (mIU/ml)		GnRH (pg/ml)		FSH (mIU/ml)	
		Before intervention	After intervention	Before intervention	After intervention	Before intervention	After intervention
Intervention group	81	14.41 ± 6.73	12.33 ± 5.51	33.32 ± 34.36	40.73 ± 33.62	5.52 ± 1.33	4.55 ± 2.41
Control group	82	15.08 ± 5.81	14.02 ± 8.62	33.68 ± 23.51	34.27 ± 23.45	6.63 ± 1.65	6.53 ± 3.72
*t*		0.681	4.133	0.078	1.424	4.725	4.028
*P*		>0.05	<0.05	>0.05	>0.05	>0.05	<0.05

**Table 9:** Changes in E2 and P indexes in the luteal phase before and after glucose supplement intervention [$\bar{x}\pm s$].

Group	*N*	E2 (pg/ml)		*P* (ng/ml)	
		Before intervention	After intervention	Before intervention	After intervention
Intervention group	81	134.42 ± 81.73	107.98 ± 48.36	6.73 ± 7.22	8.76 ± 5.14
Control group	82	133.45 ± 81.05	98.45 ± 64.27	6.58 ± 7.15	7.09 ± .1.98
*t*		0.076	1.765	0.133	2.743
*P*		>0.05	>0.05	>0.05	<0.05

The article "Multifactor Analysis and Intervention Study on Menstrual Disorders of Female Athletes in the Context of the Winter Olympic Games: A Case-Control Study Based on a Large Sample" was retracted in 2023. Reasons: unreliable results or conclusions; concerns about the data; concerns about the results or conclusions; concerns about the peer review.

## Data Availability

The data sets used and analyzed during the current study are available from the corresponding author upon reasonable request.
